# Improvement of Chloride Transport Defect by Gonadotropin-Releasing Hormone (GnRH) in Cystic Fibrosis Epithelial Cells

**DOI:** 10.1371/journal.pone.0088964

**Published:** 2014-02-19

**Authors:** Nathalie Benz, Sophie Le Hir, Caroline Norez, Mathieu Kerbiriou, Marie-Laure Calvez, Frédéric Becq, Pascal Trouvé, Claude Férec

**Affiliations:** 1 Institut National de la Santé et de la Recherche Médicale, UMR1078, Brest, France; 2 Association Gaetan Saleun, Brest, France; 3 C.H.U. Brest, Hôpital Morvan, Laboratoire de Génétique Moléculaire, Brest, France; 4 Institut de Physiologie et Biologie Cellulaires, Centre national de la recherche scientifique FRE 3511, Université de Poitiers, Poitiers, France; 5 Université de Bretagne Occidentale, Faculté de Médecine et des sciences de la santé, Brest, France; 6 Etablissement Français du Sang - Bretagne, Brest, France; University of Tübingen, Germany

## Abstract

Cystic fibrosis (CF), the most common autosomal recessive disease in Caucasians, is due to mutations in the CFTR gene. F508del, the most frequent mutation in patients, impairs CFTR protein folding and biosynthesis. The F508del-CFTR protein is retained in the endoplasmic reticulum (ER) and its traffic to the plasma membrane is altered. Nevertheless, if it reaches the cell surface, it exhibits a Cl^−^ channel function despite a short half-life. Pharmacological treatments may target the F508del-CFTR defect directly by binding to the mutant protein or indirectly by altering cellular proteostasis, and promote its plasma membrane targeting and stability. We previously showed that annexine A5 (AnxA5) directly binds to F508del-CFTR and, when overexpressed, promotes its membrane stability, leading to the restoration of some Cl^−^ channel function in cells. Because Gonadotropin-Releasing Hormone (GnRH) increases AnxA5 expression in some cells, we tested it in CF cells. We showed that human epithelial cells express GnRH-receptors (GnRH-R) and that GnRH induces an AnxA5 overexpression and an increased Cl^−^ channel function in F508del-CFTR cells, due to an increased stability of the protein in the membranes. Beside the numerous physiological implications of the GnRH-R expression in epithelial cells, we propose that a topical use of GnRH is a potential treatment in CF.

## Introduction

Cystic fibrosis (CF) is the most common autosomal recessive disease in Caucasians. It is caused by mutations in the gene encoding the cystic fibrosis transmembrane conductance regulator (CFTR) protein [1]. CFTR which is a member of the ATP-binding cassette (ABC) transporter superfamily, functions as an ion channel [1], [2]. It is mostly expressed in the apical membrane of epithelial cells and helps to maintain the fluid and electrolyte balance across the cell membrane. CFTR comprises two membrane-spanning domains (MSDs), two nucleotide-binding domains (NBDs) and a regulatory domain (RD). The CFTR protein undergoes a complex biosynthetic pathway in the endoplasmic reticulum (ER) in which molecular chaperones and co-chaperones are involved [3]. Wild-type CFTR (Wt-CFTR) biogenesis initiates in the ER where the protein is core-glycosylated, leading to an immature precursor form known as band B (∼145 KDa). It further undergoes maturation and glycosylation through the Golgi, originating a complex mature form (band C, ∼170-kDa) [4]. Only 25% to 70% of the precursor Wt-CFTR matures, depending on the cell type [5]. The remaining part undergoes ubiquitination and degradation by the proteasomal pathway [6], [7]. In membranes, once phosphorylated by protein kinase A (PKA) in the R domain, CFTR functions as an ATP-gated chloride (Cl^−^) channel [8].

Among the 1930 described mutations in the CFTR gene (http://www.genet.sickkids.on.ca/cftr/app), the deletion of phenylalanine at position 508 (F508del) is the most common one, associated with ∼70% of CF alleles [9]. The F508del mutation causes a protein folding defect, the nascent protein beeing retained in the ER. As a result, most of the F508del-CFTR channels are degraded intracellularly and very little is targetted to the plasma membrane [10]–[13]. Nevertheless, in the plasma membrane it exhibits a Cl^−^ channel activity despite an open probability 15 times lower than that of Wt-CFTR [14]–[16]. Furthermore, the F508del-CFTR protein has a faster turnover at the cell surface than Wt-CFTR [17].

In order to overcome the F508del-CFTR defects and provide a potential treatment for CF, potentiators aimed to correct the channel’s activity and correctors of the F508del-CFTR trafficking defect have been developed. Potentiators that increase the mutated CFTR’s channel activity when it is phosphorylated function via direct binding to modulate the NBDs dimerization or to increase ATP binding and hydrolysis [18]–[20]. Correctors may act indirectly or by a direct binding to F508del-CFTR. Indirect correctors such as 4-phenylbutyrate [21], glycerol [22], low temperature [23] and miglustat [24] act upon folding, ER retention, degradation and F508del-CFTR trafficking. To date, only few correctors that act specifically on F508del-CFTR by a direct binding and called pharmacological chaperones, are reported. These are VRT325, Corr4a, VRT532 and benzo[*c*]quinolizinium compounds [25]–[27]. Among potential proteins that bind to CFTR, we demonstrated that annexin A5 (AnxA5) binds directly to Wt- and F508del-CFTR when the channel is in the plasma membrane of cells. Indeed, we showed that AnxA5 is associated with the NBD1 of CFTR and using a siRNA and overexpression approach, we showed that CFTR’s channel function and membrane localization were dependent on AnxA5 expression [28].

Because our previous results showed that raised AnxA5 expression induced an augmented function of F508del-CFTR due to increased membrane localization [29], the aim of the present study was to highlight a mean to increase AnxA5 expression in F508del-CFTR expressing cells, using a drug with no side effect upon cell survival. Because it was previously showed that AnxA5 is synthesized in gonadotropes and in various cell types under the effect of gonadotropin-releasing hormone (GnRH) or some of its analogs, through mitogen activated protein kinase (MAPK), we tested the hypothesis that GnRH could increase AnxA5 expression in a human epithelial cell line and subsequently induce an increased F508del-CFTR function [30]–[32]. Using PCR, western blottings, iodide (I^−^) efflux experiments and patch-clamp experiments we show here that human epithelial cells express GnRH- receptors (GnRH-R) and that GnRH induces an AnxA5 overexpression and subsequently an increased Cl^−^ channel function of F508del-CFTR, likely due to an increased localization of the protein in membranes.

In conclusion, we show here that human epithelial cells do express GnRH-R, which has numerous physiological implications. We also propose that a topical use of GnRH is a potential treatment for CF.

## Methods

### Cell Culture

The 16HBE14o^−^ and the CFBE41o^−^ airway epithelial cell lines were obtained from Professor D. Gruenert [33], [34]. The 16HBE14o− cell line was originally developed from human bronchial epithelium to study CFTR and retains many features of differentiated bronchial epithelial cells [33]. The CFBE41o- respiratory epithelial cell line was derived from the bronchus of a patient with cystic fibrosis and immortalized with SV40. Cell culture media and supplements were purchased from Lonza (Basel, Switzerland) and PAA (Pasching, Austria). The transduced CFBE41o^−^ cell lines (CFBE41o^−/^corrected called CFBE41o−/corr and CFBE41o^−/^F508del) used in experiments were cultured as described previously [35]. CFBE41o^−/^corr and CFBE41o^−/^F508del cells were obtained by wild-type and F508del-CFTR cDNA stably introduction into CFBE41o^−^ cells, harbouring therefore the same genetic background [34], [36]. Cells were treated with 10^−9 ^M synthetic GnRH ([Gly-OH10]-LH-RH) from Sigma-Aldrich (Saint-Louis, MO, USA) for 30, 60, 120, 180 and 310 min.

### Transfection

For GnRH-R overexpression and inhibition, cells were transfected using Lipofectamine 2000 (Life Technologies Corporation, Carlsbad, CA, USA), according to the manufacturer’s instructions, with either the human cDNA clone pCMV6-XL5/GNRH-R (OriGene Technologies Inc., Rockville, MD, USA) or the human GnRH-R siRNA (5′-GGAAUUUGGUAUUGGUUUG-3′, siGENOME individual duplex (Thermo Fisher Scientific Inc., Waltham, MA, USA). The scrambled control siRNA was siGENOME Non-Targeting (Thermo Fisher Scientific Inc.).

### RNA Extraction and Quantitative Real-time PCR

Quantitative Real-Time PCR was performed to assess the basal GnRH-R and AnxA5 mRNA expression in cells and to study their modulation after GnRH treatment. Cultured medium was removed and cells were washed twice with phosphate-buffered saline (PBS). RNA was extracted using RNeasy Plus mini kit (QIAGEN, Mississauga, ON, Canada) according to the manufacturer’s instructions. Extracted RNA was eluted in RNase-free water and the concentration was determinated using a nano-photometer (Implen GmbH, München, Germany). Relative quantification of the transcripts was assessed in a two steps format (RT and qPCR). Real-Time PCR was performed using a QuantiTect® SYBR® Green PCR kit (QIAGEN, Mississauga, ON, Canada), according to the manufacturer’s instructions. A Chromo 4™ System (Bio-Rad Laboratories Inc., Hercules, CA, USA) was used to amplify cDNAs and detect emitted fluorescence. The following primers were used: GnRH-R (319 pb), forward 5′-GACCTTGTCTGGAAAGATCC-3′ and reverse 5′-CAGGCTGATCACCACCATCA-3′; AnxA5 (149 pb), forward 5′-TTCTCAGAGGCACTGTGACTGACT-3′ and reverse 5′-GATTTCCTGGCGCTGAGCATTACT-3′; G3PDH (121 pb), forward 5′-CCCATGTTCGTCATGGGTGTGAAC-3′ and reverse 5′-CAAAGTTGTCATGGATGACCTTGGC-3′. Reactions were carried out with the following parameters: enzyme activation at 95°C for 15 min, denaturation at 95°C for 30 sec, annealing at 57°C for 30 sec, extension at 72°C for 30 sec and a final extension at 72°C for 10 min. 30 and 35 cycles were used for AnxA5 and GnRH-R, respectively. For negative controls (NTC), cDNA was replaced by sterile RNase free water. Poly-A^+^ mRNA from human breast adenocarcinoma (MCF 7 cells) and Poly-A^+^ mRNA from human pituitary gland (both from Clontech, Member of Takara Bio Inc., Shigan, Japan**)** were used as positive controls.

### Protein Extraction and Western Blot Analysis

Untreated cells and GnRH treated cells were washed twice with cold PBS and were lyzed in RIPA buffer (25 mM Tris, 150 mM NaCl, 1% Triton X-100, 1% Na-Deoxycholate, 0.1% SDS, 10 mM iodoacetamide, 100 µM PMSF; pH = 7.5) in the presence of Complete Protease Inhibitor Cocktail (Roche, Basel, Switzerland). Total protein concentrations were determined using Lowry’s methodology using bovine serum albumin as a standard [37]. Samples were resolved by SDS-PAGE (7.5 to 10%) and transferred onto a PVDF membrane (GE Healthcare, Chalfont St Giles, UK). After blotting, membranes were blocked with 5% (w/v) non-fat dried skimmed milk in PBS-0.1%Tween 20 or TBST (Tris-buffered saline plus 0.1% Tween 20). Blots were probed overnight at 4°C with mouse monoclonal antibody anti-GnRH-R (1∶150, LH-RH Receptor Ab-3, clone GNRH03, MM France, Francheville, France) or goat polyclonal antibody anti-AnxA5 (1∶400, clone R-20, Santa Cruz Biotechnology, CA, USA). Blots were further incubated with HRP-conjugated secondary antibodies [1∶20000, anti-mouse and anti-goat secondary antibody were from Santa Cruz Biotechnology and Abcam (Cambridge, UK), respectively] and visualized by enhanced chemiluminescence. ECL Plus and Forte chemiluminescence detection kits were from GE Healthcare and Merk Millipore (Billerica, MA, USA), respectively. The relative intensity of each band was estimated by densitometry using BIO-1D software (BioRad). Each value was normalized to the amount of G3PDH in the same lane which was assessed on the same immunoblots probed with mouse monoclonal antibody anti-G3PDH (1∶30000, clone 6C5, Interchim SA, Montluçon, France). Positive controls for GnRH-R and AnxA5 were a whole cell lysates of human breast duct carcinoma (T-47D, Tebu-Bio, Le-Perray-en-Yvelines, France) and pure AnxA5 from human placenta (33 kD, Sigma-Aldrich), respectively.

### I^−^ Effluxes Experiments

Cells were cultured in 24-well microplates for 3 to 7days. Confluent monolayers were used, and iodide effluxes were assayed as previously described [38]. Briefly, the F508del-CFTR Cl^–^ channel activity was assayed by measuring the rate of iodide (^125^I) efflux from cells and time-dependent rates of ^125^I efflux were calculated from the following: ln (^125^I t1/^125^It2)/(t1– t2), where ^125^It is the intracellular ^125^I at time t, and t1 and t2 successive time points. Curves were constructed by plotting rates of ^125^I versus time. All comparisons were based on maximal values for the time-dependent rates (k = peak rates, min^–1^), excluding the points used to establish the baseline (k peak-k basal, min^–1^). Activators were included in the efflux buffer from time 3 min, and collection continued at 1-min intervals for an additional 7 min in the continued presence of tested compounds (for other details, [38])). To test the effect of GnRH exposure on halide permeability, CF and non-CF cells monolayers were incubated with 0.1 to 100 nM GnRH for 1 h before the efflux experiment.

### Patch-clamp Experiments

Patch-clamp experiments were performed with an automatic Nanion’s electrophysiology workstations Port-a-Patch (Nanion Technologies GmbH, Germany) coupled to an external amplifier unit HEKA EPC-10 [39]. Whole-cell patch-clamp recordings were performed at room temperature (20–25°C) on isolated CFBE41o−/corr and CFBE41o−/F508del cells, with and without GnRH treatment. Before recording, the culture medium was replaced by the external solution contained the following (in mM): 140 NaCl, 2 CaCl2, 1 MgCl2, 10 Hepes, 5 D-glucose monohydrate. Its final pH value was adjusted to 7.4 with NaOH and its osmolarity was 298 mOsmol. The internal solution contained the following (in mM): 50 CsCl, 10 NaCl, 60 Cs-Fluoride, 20 EGTA, 10 Hepes/CsOH, and 5 Mg-ATP (Mg salt); pH 7.2; 285 mOsmol. CFTR-inhibitor solution (10 µM CFTRinh172, Sigma) and CFTR-activator solution (10 µM forskolin and 30 µM genistein both from Sigma) were added to the external solution to inhibit or activate CFTR, respectively. Voltage-clamp pulses were generated and data were captured using the Patchmaster program (Nanion Technologies GmbH, Germany). Voltage-dependent properties were assessed by applying voltage steps of 100 ms duration from a holding potential of - 80 mV to test potentials ranging from −80 to +80 mV with 10 mV increments. Series resistance was compensated. For graphic representations of I/V relationship currents were normalized by membrane capacitances to remove variability due to differences in cell sizes.

### Cell Surface Biotinylation

Cells were grown in serum-free medium overnight before GnRH incubation. Culture medium was then removed and cells were washed three times with PBS plus 0.1 mM CaCl2 and 1 mM MgCl2 (pH 7.4) and once with PBS (pH 8). Cells were exposed to sulfo-NHS-SS-biotin for 30 min on ice, rinsed twice with BSA quenching buffer (1% BSA in PBS, pH 7.4) and incubated 10 min in the same buffer. Cells were scraped in PBS, pH 7.4 and centrifuged at 2400 rpm (6 min, 4°C). Cell pellets were suspended in RIPA buffer plus anti-proteases and incubated for 30 min on ice. The resulting lysates were centrifuged at 16000 g for 15 min at 4°C and total cellular protein content was determined using Lowry’s method. The supernatants were incubated with streptavidin beads (Novagen/EMD Chemicals, Madison, WI, USA) overnight at 4°C. After a brief centrifugation, supernatants were removed and the beads were washed four times in RIPA. Biotinylated proteins were eluted from streptavidin beads using 5X sample buffer containing 2-mercaptoethanol to cleave the NHS-SS-biotin and western blots were probed overnight at 4°C with a mouse monoclonal anti-CFTR antibody (1∶500, clone M3A7, Merk Millipore). For normalization, Na^+^/K^+^-ATPase expression was assessed on the same blots probed with a mouse monoclonal antibody (1∶200, clone 9-A5, Santa Cruz Biotechnology). A positive control was used to assess the mature band of CFTR (T84, human colorectal carcinoma whole cell lysate).

### Confocal Microscopy

CFBE41o^−/^corr and CFBE41o^−/^F508del cells were plated on 18-mm diameter glass coverslips at low density and maintained in culture at 37°C for 24 to 48 h before exposure to GnRH. Cells were rinsed in TBS, fixed (3% paraformaldehyde in TBS, 20 min, room temperature), rinsed in TBS, permeabilized (0.10% Triton X-100 in TBS) and rinsed again. The samples were then stained by indirect immunofluorescence. After fixation, non-specific sites were blocked with 0.5% bovine serum albumin (BSA) in TBS (60 min at room temperature). The cells were then stained with primary antibody (anti-CFTR antibody 24-1, 1∶50, RD Systems, Minneapolis, MN, USA) for 90 min at room temperature and rinsed four times in TBS containing 0.5% BSA. Next, samples were incubated with the goat anti-mouse secondary antibody conjugated to Cy3 (1∶400, Jackson Immunoresearch Laboratories, West Grove, PA, USA) for 60 min at room temperature. After final washes, samples were mounted in VectaShield plus DAPI (VECTOR Laboratories Inc., Burlingame, CA, USA), dried, and viewed with a confocal laser-scanning microscope (LSM 780, Axio Observer, Plan-Apochromat 63X/1.40 oil; Carl Zeiss GmbH, Jena, Germany). Negative controls in which primary antibody was omitted was performed.

### Statistics

Results are expressed as the means ± S.E.M of n observations. Data were compared using the Student’s t test analysis with STATGRAPHICS version 4.1 (SIGMA PLUS, Levallois-Perret, France) and differences were considered statistically significant when p<0.001 (***); p<0.01 (**) and p<0.05 (*).

## Results

### Basal Expression of GnRH-R

Basal mRNA and protein expression of GnRH-R was assessed in 16HBE14o^−^, CFBE41o^−^, CFBE41o^−/^corr and CFBE41o^−/^F508del cells. As shown in Fig. 1A, a single PCR band for GnRH-R (319 bp) was observed in the four cell lines whereas no signal was observed in the negative control. cDNAs from human pituitary gland and human MCF7 cell line (breast adenocarcinoma), were used as positive controls. The mRNA expression of G3PDH (121 bp) in the same samples showed no variation of the signal intensity. The mRNA expression of GnRH-R was quantified (Fig. 1B). Because the genetic background is only comparable between CFBE41o−/corr and CFBE41o−/F508del cells, statistical analysis was only performed for these cells and a higher mRNA expression was observed in CFBE41o−/F508del cells. Western blots were performed to detect GnRH-R (64 kDa) and G3PDH (37 kDa) in the cell lines (Fig. 1C), using a whole cell lysate of human breast duct carcinoma (T -47D) as a control. The results indicate that the GnRH-R is present in all the samples. The densitometric analysis of the signals (Fig. 1D) did not show any difference between CFBE41o−/corr and CFBE41o−/F508del cells.

**Figure 1:** Basal mRNA and protein expression of GnRH-R. **A.** The upper left panel shows representative PCR bands for GnRH-R (319 bp) after separation (2% agarose gel). A single band is observed in 16HBE14o^−^ (lane 1), CFBE41o^−^ (lane 2), CFBE41o^−/^corr (lane 3) and CFBE41o^−/^F508del (lane 4) cells. No signal is observed in the negative control (lane 5). The upper right panel shows positive controls (human pituitary gland and human MCF7cell line, lanes 1 and 2, respectively) for the detection of GnRH-R. cDNAs were from the human pituitary gland and the human MCF7cell line (breast adenocarcinoma), respectively. The mRNA expression of G3PDH (121 bp) is shown lower panel for the same samples. MW is the molecular weight given in base pairs (bp). **B.** The quantitative analysis (n = 5) of the mRNA of GnRH-R. Ct is the Cycle Threshold. A hight Ct correspond to **low mRNA** abundance because more PCR cycles are needed to detect it. Endogenous control has a lower Ct than the target mRNA. Therefore, a low ΔCt ( = Ct gene – Ct control) correspond to high mRNA abundance **C.** Upper panel shows representative immunoblots of GnRH-R (64 kDa) and lower panel shows representative immunoblots of G3PDH (37 kDa). A protein expression is observed in 16HBE14o^−^ (lane 1), CFBE41o^−^ (lane 2), CFBE41o^−/^corr (lane 3) and CFBE41o^−/^F508del (lane 4) cells. A positive control (lane 5) was used for the detection of GnRH-R (human breast duct carcinoma (T-47D) whole cell lysate). G3PDH was used for further normalization. **D.** The densitometric analysis of GnRH-R expression (n = 6) did not show any difference between cell lines.

To assess the GnRH-R antibody’s specificity, the GnRH-R’s expression was modulated before immunodetection. First, 16HBE14o^−^, CFBE41o^−^ cells were transfected with a GnRH-R expression vector in which the cDNA encoding GnRH-R was ligated. As shown in Fig. 2A, the immunoblots indicated that the transfection induced an increased expression of the receptor. The control cells were transfected with the empty vector and G3PDH was detected for further normalization. The quantitative analysis of the blots (Fig. 2B) showed that the transfection of the expression vector induced an increased expression of GnRH-R of 70% and 44% in 16HBE14o^−^, CFBE41o^−^ cells, respectively, when compared to the control cells. Second, a siRNA directed against GnRH-R was used and a decreased expression of the protein was observed in both cell types (Fig. 2C). The quantitative analysis of the blots (Fig. 2D) showed that the siRNA induced an decrease expression of GnRH-R of 64% and 65% in 16HBE14o^−^, CFBE41o^−^ cells, respectively, when compared to the control cells which were transfected with a scrambled siRNA.

**Figure 2:** Validation of the detection of GnRH-R in immunoblots. **A.** Representative immunoblots of GnRH-R detection (upper panel) after 48 h transfection with the Human cDNA clone pCMV6-XL5/GNRH-R in 16HBE14o^−^ (1) and CFBE41o^−^ (2) cells. pCMV6-XL5 empty plasmid was used as a control. **B.** The densitometric analysis after normalization by G3PDH expression and comparison with the controls, indicate that the GnRH-R expression in significantly increased, (n = 5). **C.** Representative immunoblots of GnRH-R detection after 72 h transfection with a siGENOME individual duplex targeting GnRH-R in 16HBE14o^−^ (1) and CFBE41o^−^ (2) cells. siGENOME Non-Targeting was used as control. A decreased expression of GnRH-R is observed in both cell types. **D.** The densitometric analysis after normalization by G3PDH expression and comparison with the controls, indicate that the GnRH-R expression is significantly decreased in 16HBE14o^−^ (1) and CFBE41o^−^ (2) cells (n = 7) in the presence of siRNA.

### Basal Expression of AnxA5

Basal mRNA and protein expression of AnxA5 was assessed in 16HBE14o^−^, CFBE41o^−^, CFBE41o^−/^corr and CFBE41o−/F508del cells. As shown in Fig. 3A, AnxA5 mRNA (149 bp) was detected in all cell lines whereas, no signal was observed in the negative control. The gene expression of AnxA5 was quantified in cells using Real-Time PCR. Analysis of the data (Fig. 3B) between CFBE41o−/corr and CFBE41o−/F508del cells showed a higher expression in the cells expressing the mutated CFTR. AnxA5 expression was further assessed by western blottings (Fig. 3C). The statistical analysis (Fig. 3D) indicated that AnxA5 expression does not vary within cell lines. Nevertheless, the amount of AnxA5 protein tended to be higher in CFBE41o−/corr and CFBE41o^−/^F508del cells than in 16HBE14o^−^ or CFBE41o^−^ cells.

**Figure 3:** Basal mRNA and protein expression of AnxA5. **A.** The left image shows representative PCR bands for AnxA5 (149 bp) and the right image shows representative PCR bands for G3PDH (121 bp, 2% agarose gel). A single band is observed in 16HBE14o^−^ (lane 1), CFBE41o^−^ (lane 2), CFBE41o^−/^corr (lane 3) and CFBE41o^−/^F508del (lane 4) cells. No signal is observed in the negative control (lane 5). MW is the molecular weight given in base pairs (bp). B. The gene expression of AnxA5 was determined by quantitative Real-Time PCR in each cell line and data were analyzed by using ΔCt (target – reference). Comparison between CFBE41o^−/^corr (3) and CFBE41o^−/^F508del (4) cells show a higher expression in CF cells. C. The upper image shows a representative immunodetection of AnxA5 protein (35 kDa) and the lower image shows the immunodetection of G3PDH (37 kDa) protein expression in 16HBE14o^−^ (lane 1), CFBE41o^−^ (lane 2), CFBE41o^−/^corr (lane 3) and CFBE41o^−/^F508del (lane 4) cells. Pure AnxA5 was used as a positive control (lane 5). G3PDH was detected to show that the loading was identical in each lane and for further normalization. D. Statistical analysis of AnxA5 expression (n = 6) indicate that the expression of AnxA5 does not vary among cell lines although it tends to be higher in CFBE41o^−/^corr and CFBE41o^−/^F508del cells than in 16HBE14o^−^ or CFBE41o^−^ cells.

### AnxA5 Expression in Cells Submitted to GnRH Treatment for 60 min

In order to determine whether GnRH modulates AnxA5 expression and to determine the shortest time to be used for GnRH treatment, 16HBE14o^−^, CFBE41o^−^, CFBE41o^−/^corr and CFBE41o^−/^F508del cells were treated with 10^−9 ^M GnRH for 30, 60, 120, 180 and 310 min (not shown). At each time point, the protein expression of AnxA5 was evaluated and normalized with that of G3PDH. The AnxA5 expression was compared to that of cells incubated with buffer alone used as a control. Fig. 4A shows an example of the obtained western blots at the 60 min time point. An increased intensity of the AnxA5 band was observed in all cell types. Densitometry of the bands, normalization using G3PDH and quantification were performed (Fig. 4B). It was concluded that a 60 min treatment led to a significant increase of AnxA5 expression in the four cell types.

**Figure 4:** AnxA5 expression when cells are treated for 60 min with GnRH. **A.** Representative immunoblots showing AnxA5 and G3PDH expression in 16HBE14o^−^ (1), CFBE41o^−^ (2), CFBE41o^−/^corr (3) and CFBE41o^−/^F508del (4) cells after 60 min of treatment by GnRH (10^−9^ M). An increased expression is observed in all cell types. **B.** Densitometric analysis of AnxA5 expression. Data are normalized by G3PDH. AnxA5 protein expression is presented as mean ± S.E.M (7 independent experiments with n ≥2 for each experiment). For each cell line, the statistical analysis was performed by comparing the normalized amount of AnxA5 between cells incubated with buffer alone (white bars adjusted to 1) and cells incubated with GnRH (black bars).

### Increased Endogenous F508del-CFTR’s Function by GnRH Treatment

To test the activity of CFTR channels under GnRH treatment in 16HBE14o^−^, CFBE41o^−^, CFBE41o^−/^corr and CFBE41o^_^/F508del cells, functional analysis was performed by measuring the cAMP regulated and CFTR-dependent iodide efflux after 1 h incubation at 37°C with GnRH (10^−9^ M). The activity of CFTR was stimulated by a mixture of adenylate cyclase activator forskolin (Fsk, 10 µM) plus isoflavone genistein (Gst, 30 µM) or inhibited by the thiazolidinone specific CFTR blocker CFTRinh-172 (10 µM). Example of mean traces showing an increased iodide efflux in 16HBE14o^−^ cells, untreated or treated with GnRH is shown in Fig. 5A. This example shows that after adding Fsk/Gst, the rate of iodide efflux increased at a maximum rate (peak value) after 4 min and that the peak was higher in the presence of GnRH. Experiments were conducted for all cell types and the results are represented as bar graphs in Fig. 5B. Statistical analysis indicated that in the presence of GnRH, the rates of iodide efflux were significantly increased in 16HBE14o^−^, CFBE41o^−^, CFBE41o^−/^corr and CFBE41o^−/^F508del cells when compared to untreated cells, indicating that CFTR and F508del-CFTR’s function are increased by GnRH. The concentration-response effect of GnRH was further determined in the presence or absence of Fsk and Gst (Fig. 6). Calculated an EC50 in 16HBE14o^−^, CFBE41o^−^, CFBE41o^−/^corr and CFBE41o^−/^F508del cells were 0.6±1.4 nM, 0.8±1.2 nM, 0.9±1.3 nM and 2.2±1.4 nM, respectively.

**Figure 5:** Activation of wild-type and F508del-CFTR chloride channel activity in cells treated by GnRH. **A.** Example of mean traces showing the restoration of an iodide efflux in 16HBE14o- cells untreated or treated 1 h with 1 nM GnRH and stimulated by 10 µM forskolin and 30 µM genistein. **B.** Bar graph showing the enhancement of the chloride channel function of CFTR in 16HBE14o^−^, CFBE41o^−^, CFBE41o^−/^corr and CFBE41o^−/^F508del cells (1, 2, 3 and 4, respectively) using iodide efflux experiments. Histograms show the mean relative rate of iodide efflux in each cell type, with and without GnRH treatement. A significant increase is observed in the presence of GnRH (n = 4).

**Figure 6:** Concentration-dependent effect of GnRH. Concentration-dependent enhancement of CFTR’s function by GnRH in 16HBE14o^−^ (A), CFBE41o^−^ (B), CFBE41o^−/^corr (C) and CFBE41o^−/^F508del (D): CFTR activity was assessed with the iodide effluxes technique in the presence of forskoline (10 µM) plus genistein (30 µM) after 1h of incubation. Results are expressed as normalized means (± SEM, n = 4).

CFTR’s function in CFBE41o−/corr and CFBE41o_/F508del cells was also assessed by patch-clamp experiments in the whole cell configuration ((n = 5 to 9 cells from different cell cultures, Fig. 7). Mean cell capacitances were 21.4 and 18.66 pF for CFBE41o−/corr and CFBE41o_/F508del cells, respectively. Fig. 7A (upper panel) show the normalized I/V curve obtained when CFBE41o−/corr cells were treated or not with GnRH for 1 hour, with activators and with the CFTR inhibitor. It can be observed that activation and inhibition were efficient in both cases showing the specificity of the recordings. It was also observed that GnRH treatment of the cells induced an increased current density. Statistical analysis was further performed and presented as a bar graph (Fig. 7A, lower panel). In untreated cells inhibition and activation of CFTR were significantly efficient whereas in treated cells only inhibition led to a significant decreased current density. When untreated cells were compared to treated cells, solely the basal current densities were significantly increased by GnRH. The absence of activation by Fsk/Gst in GnRH treated cells could be explained by the fact that the concentration of the activators was the same in both treated and untreated cells and because the basal current density was higher in the presence of GnRH. The drawn conclusion is that GnRH induces an increased current density in CFBE41o−/corr cells. I/V curves obtained with CFBE41o_/F508del cells in the same conditions as for CFBE41o−/corr cells are shown in Fig. 7B (upper panel). As in Fig. 7A, basal normalized currents, as well as modulated currents by activation and inhibition were higher in the presence of GnRH. Statistical analysis and bar graphs (Fig. 7B, lower panel) showed a basal current in untreated CFBE41o_/F508del cells, likely due to the presence of Mg-ATP in the internal solution, activating the weak quantity of CFTR within membranes. The use of Fsk/Gst and CFTRinh-172 was inefficient upon the mutated CFTR’s function. In treated cells, the basal current density was close to 5 times higher than in untreated cells. This difference was highly significant despite being lower than in CFBE41o−/corr cells. In these conditions, Fsk/Gst and CFTRinh-172 were efficient as in corrected cells. Therefore, F508del-CFTR’s function under GnRH treatment exhibited the same pattern as Wt-CFTR, with a much lower intensity (in the range of 100 pA).

**Figure 7:** Activation of CFTR current in CFBE41o−/corr and CFBE41o−/F508del cells by patch –clamp experiments. **A.** Upper panel shows I/V curves (normalized by cell capacitance pF, mean±SEM) for CFTR current in CFBE41o−/corr cells in the whole cell configuration. Basal condition is with MgATP in the intracellular buffer. CFTR was activated by forskolin plus genistein and inhibited by CFTR inhibitor 172. Curves obtained with and without GnRH treatment (1 hour) were plotted. The lower panel shows the statistical analysis of the currents noted at +80 mV. **B.** Same as in A for CFBE41o−/F508del cells.

### Increased Membrane Expression of CFTR after GnRH Treatment

The presence of CFTR within membranes after 1 hour treatment by GnRH was assessed by biotinylation experiments. Cells were biotinylated with Sulfo-NHS-SS-biotin, pulled-down with streptavidin-agarose and subjected to 7.5% SDS-PAGE. Total cell lysates were used as controls. Representative immunoblots showing the detection of CFTR in biotinylated surface proteins from 16HBE14o^−^ and CFBE41o^−/^corr cells are shown in Fig. 8A and 8B, respectively. CFTR was present in total lysates and in pulled down samples. The densitometric analysis of CFTR’s cell surface expression was performed and normalized with the biotinylated Na^+^/K^+^-ATPase level. The statistical analysis clearly indicates that the amount of biotinylated CFTR is higher after GnRH treated cells (Fig. 8C). An increased amount of CFTR in membranes of 33 and 36% was observed in 16HBE14o^−^ and CFBE41o^−/^corr cells, respectively. Whereas CFTR was detected in controls, we failed to detect it in biotinylated surface proteins from CFBE41o^−^ and CFBE41o^−/^F508del cells (not shown).

**Figure 8:** Membrane expression of CFTR after GnRH treatment. The presence of CFTR within membranes was detected by biotinylation experiments. **A.** Representative immunoblots showing the detection of CFTR in biotinylated surface proteins from 16HBE14o^−^ cells. CFTR is present in total proteins (left) and in biotinylated surface proteins (right) after GnRH treatment (10^−9^ M) for 60 min. The arrowheads indicate the fully glycosylated (180 kDa) CFTR. B. Same image as in A. with CFBE41o^−/^corr cells. C. Histograms of the densitometric analysis of CFTR’s cell surface expression (n = 4) in 16HBE14o^−^ (1) and CFBE41o^−/^corr (2) cells The biotinylated CFTR level is normalized to the biotinylated Na^+^/K^+^-ATPase level. Cells incubated with buffer alone are referred as 1 arbitrary unit.

### Increased Membrane Localization of CFTR after GnRH Treatment

Because we failed to detect CFTR in CFBE41o^−^ and CFBE41o^−/^F508del cells due to the poor expression of the protein, membrane localization of CFTR in CFBE41o^−/^F508del cells was assessed by confocal microscopy, in the absence (Fig. 9A) and in the presence (Fig. 9B) of a GnRH treatment (120 min). Without any treatment, CFTR was mainly observed around the nuclei of the cells. We therefore speculated that it was present in the ER. When cell were treated with GnRH, CFTR had a more spread localization and it was observed at the periphery of the cells, looking like the plasma membrane, as shown in Fig. 9B by white arrows. Controls performed without CFTR antibody showed no labelling (not shown).

**Figure 9:** Immunolocalization of CFTR in CFBE41o−/F508del cells after GnRH treatment. A. Representative confocal photomicrographs of the localization of F508del-CFTR in cells without any treatment. CFTR is likely observed around the nuclei, in the endpoplasmic reticulum. B. Representative confocal photomicrographs of the localization of F508del-CFTR in cells after GnRH treatment. CFTR is likely observed in the endpoplasmic reticulum but also in membranes.

### Comparison of the Effect of Miglustat and GnRH

The time-dependent effects of miglustat and GnRH were assessed and compared in CFBE41o^−^ and CFBE41o^−/^F508del cells (Fig. 10). CFTR’s function was assessed by the iodide effluxes technique in the presence of 1 nM GnRH or 100 µM miglustat. As shown in Fig. 10A, miglustat induced an increased iodide efflux in CFBE41o^−^ cells after 1 hour treatment. The increase was higher at the 2 hours time point. GnRH also induced an increased iodide efflux but the effect was lower, but significant, and did not increase after 2 hours of treatment. In CFBE41o^−/^F508del cells (Fig. 10B), the same time-dependent effect as in CFBE41o^−^ cells was observed.

**Figure 10:** Comparison of the effect of miglustat and GnRH. Comparison of the time-dependent effect of GnRH or miglustat upon F508del-CFTR function in CFBE41o- cells (A) and in CFBE41o^−/^F508del cells (B). CFTR activity was assessed with the iodide effluxes technique in the presence of forskolin (10 µM) plus genistein (30 µM) after 1 nM GnRH or 100 µM miglustat incubation (n = 4).

## Discussion

The most common mutation causing CF, F508del-CFTR, is known for more than 20 years [1]. The F508del-CFTR nascent protein is recognized by the cellular quality control machinery and is degraded. A very small amount succeeds in trafficking to the cell membrane where it functions as a Cl^−^ channel. Many efforts were performed in order to identify molecules that could correct the trafficking defect. Indeed, it is estimated that the required correction to ameliorate the symptoms in CF patients is between 10% and 30% of wild-type CFTR function [40], [41].

Among proteins that directly bind to CFTR, we previously showed that AnxA5 binds to NBD1 and, when over expressed, may restore some Cl^−^ channel function due to an increased stabilization of CFTR in membranes [28], [29]. AnxA5 belongs to the annexin family which is characterized by calcium-dependent phospholipid binding. Annexins are found in a wide variety of species, from plants to human [42]–[44]. They are known to inhibit PLA2, PKC, and blood coagulation [42]. Under specific conditions, AnxA5 can also form a calcium channel [45]. Despite these molecular characteristics, their physiological role within cells remains unclear.

Whereas the CFTR/AnxA5 interaction as well as the augmented Wt-CFTR whole-cell currents, due to over-expression of AnxA5, was further confirmed, it was not seen in F508del-CFTR expressing cells [46]. The discrepancy with our previous results and within the referred study is likely due to the used cell system. These authors suspect that AnxA5 does not interact specifically with CFTR. This discrepancy is likely due to the use of a non specific AnxA5 antibody [46]. Because it is suggested that some CFTR is expressed at the apical membrane in epithelial cells from CF patients [47], despite a reduced level when compared to non-CF cells, and because we found a positive effect of AnxA5, our aim was to highlight a non toxic mean to increase AnxA5 expression in F508del-CFTR expressing cells. Some previous results clearly demonstrate that GnRH stimulation induces the expression of AnxA5 in the gonadotropes, luteal cells and other cell types [30]–[32]. Therefore, we tested the hypothesis of an AnxA5 increased synthesis in response to GnRH stimulation in human epithelial cells of the airways.

GnRH is secreted by GnRH neurons in the hypothalamus and is transported to the gonadotropes of the anterior pituitary gland. It is a decapeptide involved in the control of reproduction and binds to a specific G protein-coupled receptor to allow gonadotropin secretion. GnRH and its receptor are reported to be expressed in human tissues outside of the hypothalamus, such as liver, heart, skeletal muscle and kidney where its functions are unclear [48].

The first step of the present work was to assess the expression of GnRH-R and AnxA5 in human epithelial cells (Fig. 1 to 3). 16HBE14 o^−^, CFBE41o^−^ and the transduced CFBE41o^−^ airway epithelial cell lines CFBE41o^−/^corr and CFBE41o^−/^F508del were used [35]. Using PCR and western blottings, we observed an AnxA5 and GnRH-R expression in these cells. Because the genetic background of 16HBE14o^−^, CFBE41o^−^ cells are different, their GnRH-R expression was not compared. The GnRH-R expression (protein) did not vary between CFBE41o^−/^corr and CFBE41o^−/^F508del cells. Because anti-GnRH-R antibodies are debated, we decided to assure us of the results. For this, GnRH-R expression was modulated (increased and decreased) before immunodetection and we showed that the observed band was indeed GnRH-R. The GnRH-R expression in airway epithelial cells is in accordance with previous results showing its expression in extrapituitary tissues. A high expression level of the mRNA was found in prostate, thymus, and kidney. In heart, brain, placenta, lung, liver, skeletal muscle, pancreas, colon, ovary, small intestine, spleen, and testis the mRNA was also detected [49]. The presence and localization of GnRH-R in airway epithelial cells (Calu-3) was also shown using immunochemical methods [49], [50]. Here, we present for the first time the GnRH-R expression in 16HBE14o^−^, CFBE41o^−^ and the transduced CFBE41o^−^ airway epithelial cell lines, using immunoblots. AnxA5 expression was studied in our cell models at the mRNA and protein level and we found that it is also expressed. This result is in accordance with previous results [51]. Therefore, GnRH-R and AnxA5 expression being shown, further experiments were conducted.

The second step of the work was to study AnxA5 expression under GnRH treatment and the effect of the hormone on the function of CFTR (Fig. 4 to 6). The four cell types were treated with GnRH (10^−9^ M) for 30, 60, 120, 180 and 310 min (not shown) and western-blottings were performed. A significant increased AnxA5 expression was observed at the 60 min time point and remained stable until 310 min. This increased expression of AnxA5 under GnRH treatment was previously described. Indeed, a continuous exposure to GnRH driving a specific gene expression of AnxA5 without desensitization was reported [32]. Nevertheless, our further experiments were conducted at 60 min of GnRH treatment, corresponding to a significant increased AnxA5 expression in 16HBE14o^−^, CFBE41o^−^, CFBE41o^−/^corr and CFBE41o^−/^F508del cells. Functional analysis was performed by measuring the CFTR-dependent iodide efflux in the absence and in the presence of GnRH. Statistical analysis indicated that with GnRH, the rates of iodide efflux were significantly increased in 16HBE14o^−^, CFBE41o^−^, CFBE41o^−/^corr and CFBE41o^−/^F508del cells when compared to untreated cells. EC_50_ were relatively low (2.2 nM in CFBE41o^−/^F508del cells). To provide further evidence of an increased channel function of CFTR in CFBE41o−/F508del cells, whole-cell patch-clamp experiments were performed with and without GnRH treatment of the cells. The main conclusion drawn from these experiments is that in CFBE41o−/corr as well as in CFBE41o−/F508del cells, current densities via CFTR are increased in the presence of GnRH, corroborating the results obtained in iodide efflux experiments. In CFBE41o−/F508del cells, GnRH also lead to a regulation of CFTR by Fsk/Gst and CFTRinh-172, what was not observed in untreated cells. Therefore, GnRH increases sufficiently the chloride channel function of the mutated CFTR to lead to the observation of its modulation.

Our third step was to give some potential explanations to the observed increased Cl^−^ channel function of CFTR in the presence of GnRH. We assessed a possible increased anchoring of CFTR within membranes by biotinylation and confocal microscopy (Fig. 8, 9). According to our previous work [28], [29], we found that the presence of F508del-CFTR was increased in membranes. Our results showing in the CFBE41o−/F508del cells an increased CFTR membrane localization after GnRH treatment could not be related to the additional plasmid inserted in the CFBE41o- cells because in biotinylation experiments without GnRH, the amount of CFTR in 16HBE14o- cells is not different than in CFBE41o−/corr cells. Nevertheless, the observed increased Cl^−^ channel function of CFTR in the presence of GnRH is likely not only due to the weak AnxA5 overexpression. The presence of CFTR within membranes after treatment was difficult to detect and due to the pleiotropic effects of GnRH, we hypothesize that the increased AnxA5 expression in likely not the only reason for this effect. Indeed, the expression of AnxA5 is directly stimulated by GnRH, probably through protein kinase C, MAKP and calcium pathways which are also involved in the regulation and in the targeting of CFTR in membranes [30]–[32], [38], [52]–[54]. A schematic representation of our findings together with known effects of GnRH is presented in Fig. 11. The involved pathways explaining the increased membrane localization of F508del-CFTR when cells are stimulated by GnRH, as well as the involvement of calcium are under investigation in our laboratory. Interestingly, the rapid and sustained action of GnRH seems different of the action of correctors or potentiators. We found of interest to compare the action of the well known corrector miglustat [24] with that of GnRH (Fig. 10). Time dependant effects of miglustat and GnRH were different. Whereas, miglustat induced a continuous increased iodide efflux until 2 hours, the GnRH effect observed at the 1 hour time point remained stable until the 2 hours. This observation permit to say that actions are likely different and reinforce the hypothesis that GnRH does not act as a corrector. Miglustat permits F508del-CFTR to escape the ER whereas GnRH maintains it in membranes. The association of both miglustat and GnRH will be further explored in primary cultures. Nevertheless, beside miglustat, several classes of F508del-CFTR correctors have been identified and could be tested. Indeed, despite many efforts to identify potentiators (such as VX-770) and correctors (such as VX-809), and, recently, a class of compounds with dual potentiator and corrector activities, much work remain to find out new molecules with beneficial effects on F508del-CFTR defects (for review [55]). The study of a combined effect of GnRH together with recently described compounds would be of interest to assess the benefit of the association of such molecules.

**Figure 11:** Schematic representation of the GnRH’s effect on F508del-CFTR function. We found that F508del-CFTR’s membrane localization and function are increased under GnRH treatment, associated with an increased expression of AnxA5 (red lines). Nevertheless, according to previous results, AnxA5 over expression is likely not the solely event triggered in cells by GnRH. Described events are summarized in black lines and their possible involvement upon F508del-CFTR activity are shown in dotted black lines.

In conclusion, we show here for the first time that GnRH-R are expressed in the used airway epithelial cells at the protein level and we propose that GnRH restores some Cl^−^ channel function in CF cells. Because some GnRH analogs such as leuprolide, buserelin and goserelin are already used in medical practice as nasal sprays, we intend to test these medications in human primary cells.

## References

[1] RiordanJR, RommensJM, KeremB, AlonN, RozmahelR, et al (1989) Identification of the cystic fibrosis gene: cloning and characterization of complementary DNA. Science 245: 1066–1073.247591110.1126/science.2475911

[2] BearCE, LiCH, KartnerN, BridgesRJ, JensenTJ, et al (1992) Purification and functional reconstitution of the cystic fibrosis transmembrane conductance regulator (CFTR). Cell 68: 809–818.137123910.1016/0092-8674(92)90155-6

[3] AmaralMD (2004) Cftr and chaperones: Processing and degradation. J MolNeurosci 23: 41–48.10.1385/JMN:23:1-2:04115126691

[4] ChengSH, GregoryRJ, MarshallJ, PaulS, SouzaDW, et al (1990) Defective intracellular transport and processing of cftr is the molecular basis of most cystic fibrosis. Cell 63: 827–834.169966910.1016/0092-8674(90)90148-8

[5] LukacsGL, MohamedA, KartnerN, ChangXB, RiordanJR, et al (1994) Conformational maturation of cftr but not its mutant counterpart (delta f508) occurs in the endoplasmic reticulum and requires atp. EMBO J 13: 6076–6086.752917610.1002/j.1460-2075.1994.tb06954.xPMC395586

[6] JensenTJ, LooMA, PindS, WilliamsDB, GoldbergAL, et al (1995) Multiple proteolytic systems, including the proteasome, contribute to cftr processing. Cell 83: 129–135.755386410.1016/0092-8674(95)90241-4

[7] WardCL, OmuraS, KopitoRR (1995) Degradation of cftr by the ubiquitin-proteasome pathway. Cell 83: 121–127.755386310.1016/0092-8674(95)90240-6

[8] HwangTC, SheppardDN (2009) Gating of the CFTR Cl^−^ channel by ATP-driven nucleotide-binding domain dimerisation. J Physiol 587: 2151–2161.1933248810.1113/jphysiol.2009.171595PMC2697289

[9] ZielenskiJ, TsuiLC (1995) Cystic fibrosis: genotypic and phenotypic variations. Annu Rev Genet 29: 777–807.882549410.1146/annurev.ge.29.120195.004021

[10] ChengSH, GregoryRJ, MarshallJ, PaulS, SouzaDW, et al (1990) Defective intracellular transport and processing of CFTR is the molecular basis of most cystic fibrosis. Cell 63: 827–834.169966910.1016/0092-8674(90)90148-8

[11] DenningGM, AndersonMP, AmaraJF, MarshallJ, SmithAE, et al (1992) Processing of mutant cystic fibrosis transmembrane conductance regulator is temperature-sensitive. Nature 358: 761–764.138067310.1038/358761a0

[12] SatoS, WardCL, KrouseME, WineJJ, KopitoRR (1996) Glycerol reverses the misfolding phenotype of the most common cystic fibrosis mutation. J Biol Chem 271: 635–638.855766610.1074/jbc.271.2.635

[13] Welsh MJ, Denning GM, Ostedgaard LS, Anderson MP (1993) Dysfunction of CFTR bearing the delta F508 mutation. J Cell Sci. Suppl. 17: 235–239.7511616

[14] DalemansW, BarbryP, ChampignyG, JallatS, DottK, et al (1991) Altered chloride ion channel kinetics associated with the ΔF508 cystic fibrosis mutation. Nature 354: 526–528.172202710.1038/354526a0

[15] OstedgaardLS, RogersCS, DongQ, RandakCO, VermeerDW, et al (2007) Processing and function of CFTR-ΔF508 are species-dependent. Proc Natl Acad Sci USA 104: 15370–15375.1787306110.1073/pnas.0706974104PMC1976592

[16] MikiH, ZhouZ, LiM, HwangTC, BompadreSG (2010) Potentiation of disease-associated cystic fibrosis transmembrane conductance regulator mutants by hydrolyzable ATP analogs. J Biol Chem 285: 19967–19975.2040682010.1074/jbc.M109.092684PMC2888408

[17] LukacsGL, ChangXB, BearC, KartnerN, MohamedA, et al (1993) The delta F508 mutation decreases the stability of cystic fibrosis transmembrane conductance regulator in the plasma membrane. Determination of functional half-lives on transfected cells. J. Biol. Chem. 268: 21592–21598.7691813

[18] HwangTC, WangF, YangIC, ReenstraWW (1997) Genistein potentiates wild-type and delta F508-CFTR channel activity. Am. J. Physiol. 273: C988–C998.10.1152/ajpcell.1997.273.3.C9889316420

[19] CaiZ, SheppardDN (2002) Phloxine B interacts with the cystic fibrosis transmembrane conductance regulator at multiple sites to modulate channel activity. J. Biol. Chem. 277: 19546–19553.10.1074/jbc.M10802320011904291

[20] VerganiP, LocklessSW, NairnAC, GadsbyDC (2005) CFTR channel opening by ATP-driven tight dimerization of its nucleotide-binding domains. Nature 433: 876–880.1572934510.1038/nature03313PMC2756053

[21] RubensteinRC, EganME, ZeitlinPL (1997) In vitro pharmacologic restoration of CFTR-mediated chloride transport with sodium 4-phenylbutyrate in cystic fibrosis epithelial cells containing delta F508-CFTR. J. Clin. Invest. 100: 2457–2465.10.1172/JCI119788PMC5084469366560

[22] BrownCR, Hong-BrownLQ, BiwersiJ, VerkmanAS, WelchWJ (1996) Chemical chaperones correct the mutant phenotype of the delta F508 cystic fibrosis transmembrane conductance regulator protein. Cell Stress Chaperones 1: 117–125.922259710.1379/1466-1268(1996)001<0117:ccctmp>2.3.co;2PMC248464

[23] DenningGM, AndersonMP, AmaraJF, MarshallJ, SmithAE, et al (1992) Processing of mutant cystic fibrosis transmembrane conductance regulator is temperature-sensitive. Nature 358: 761–764.138067310.1038/358761a0

[24] NorezC, NoelS, WilkeM, BijveldsM, JornaH, et al (2006) Rescue of functional delF508-CFTR channels in cystic fibrosis epithelial cells by the alpha-glucosidase inhibitor miglustat. FEBS Lett. 580: 2081–2086.10.1016/j.febslet.2006.03.01016546175

[25] WangY, BartlettMC, LooTW, ClarkeDM (2006) Specific rescue of cystic fibrosis transmembrane conductance regulator processing mutants using pharmacological chaperones. Mol. Pharmacol. 70(1): 297–302.10.1124/mol.106.02399416624886

[26] WangY, LooTW, BartlettMC, ClarkeDM (2007) Correctors promote maturation of cystic fibrosis transmembrane conductance regulator (CFTR)-processing mutants by binding to the protein. J. Biol. Chem. 282: 33247–33251.10.1074/jbc.C70017520017911111

[27] BecqF, MetteyY, GrayMA, GaliettaLJ, DormerRL, et al (1999) Development of substituted Benzo[c]quinolizinium compounds as novel activators of the cystic fibrosis chloride channel. J. Biol. Chem. 274: 27415–27425.10.1074/jbc.274.39.2741510488073

[28] TrouvéP, Le DrévoMA, KerbiriouM, FichouY, GilletD, et al (2007) Annexin V is directly involved in cystic fibrosis transmembrane conductance regulator’s chloride channel function. Biochim Biophys Acta. 1772: 1121–1133.10.1016/j.bbadis.2007.06.00617869070

[29] Le DrévoMA, BenzN, KerbiriouM, GiouxM, PennecJP, et al (2008) Annexin A5 increases the cell surface expression and the chloride channel function of the ΔF508-Cystic Fibrosis Transmembrane Regulator. Biochim Biophys Acta 1782: 605–614.1877395610.1016/j.bbadis.2008.08.002

[30] KawaminamiM, EtohS, MiyaokaH, SakaiM, NishidaM, et al (2002) Annexin 5 messenger ribonucleic acid expression in pituitary gonadotropes is induced by gonadotropin-releasing hormone (GnRH) and modulates GnRH stimulation of gonadotropin release. Neuroendocrinology 75(1): 2–11.1181003010.1159/000048216

[31] YaoB, KawaminamiM (2008) Stimulation of annexin A5 expression by gonadotropin releasing hormone (GnRH) in the Leydig cells of rats. J Reprod Dev 54(4): 259–264.1850434410.1262/jrd.20039

[32] KawaminamiM, UematsuN, FunahashiK, KokubunR, KurusuS (2008) Gonadotropin releasing hormone (GnRH) enhances annexin A5 mRNA expression through mitogen activated protein kinase (MAPK) in LbetaT2 pituitary gonadotrope cells. Endocr J. 55(6): 1005–1014.10.1507/endocrj.k08e-13118703851

[33] CozensAL, YessiMJ, KunzelmannK, OhruiT, ChinL, et al (1994) CFTR expression and Chloride secretion in polarized immortal human bronchial epithelial cells. Am J Respir Cell Mol Biol 10: 38–47.750734210.1165/ajrcmb.10.1.7507342

[34] BrusciaE, SangiuoloF, SinibaldiP, GonczKK, NovelliG, et al (2002) Isolation of CF cell lines corrected at DeltaF508-CFTR locus by SFHR-mediated targeting. Gene Ther. 9: 683–685.10.1038/sj.gt.330174112032687

[35] IllekB, MaurisseR, WahlerL, KunzelmannK, FischerH, et al (2008) Cl transport in complemented CF bronchial epithelial cells correlates with CFTR mRNA expression levels. Cell. Physiol. Biochem. 22: 57–68.10.1159/000149783PMC292712018769032

[36] BebokZ, CollawnJF, WakefieldJ, ParkerW, LiY, et al (2005) Failure of cAMP agonists to activate rescued deltaF508 CFTR in CFBE41o- airway epithelial monolayers. J. Physiol. 569: 601–615.10.1113/jphysiol.2005.096669PMC146425316210354

[37] LowryOH, RosebroughNJ, FarrAL, RandallRJ (1951) Protein measurement with the Folin phenol reagent. J. Biol. Chem. 193: 265–275.14907713

[38] NorezC, AntignyF, BecqF, VandebrouckC (2006) Maintaining Low Ca2+ Level in the Endoplasmic Reticulum Restores Abnormal Endogenous F508del-CFTR Trafficking in Airway Epithelial Cells. Traffic 7: 562–573.1664327910.1111/j.1600-0854.2006.00409.x

[39] FarreC, StoelzleS, HaarmannC, GeorgeM, BrüggemannA, et al (2007) Automated ion channel screening: patch clamping made easy. Expert Opin Ther Targets 11(4): 557–65.1737388410.1517/14728222.11.4.557

[40] McKoneEF, EmersonSS, EdwardsKL, AitkenML (2003) Effect of genotype on phenotype and mortality in cystic fibrosis: a retrospective cohort study. Lancet 361: 1671–1676.1276773110.1016/S0140-6736(03)13368-5

[41] Zhang L, Button B, Gabriel SE, Burkett S, Yan Y et al. (2009) CFTR delivery to 25% of surface epithelial cells restores normal rates of mucus transport to human cystic fibrosis airway epithelium. PLoS Biol. 7 e1000155.10.1371/journal.pbio.1000155PMC270518719621064

[42] GerkeV, MossSE (2002) Annexins: from structure to function. Physiol Rev 82: 331–371.1191709210.1152/physrev.00030.2001

[43] CromptonMR, MossSE, CrumptonMJ (1988) Diversity in the lipocortin/calpactin family. Cell 55: 1–3.297145010.1016/0092-8674(88)90002-5

[44] MossSE, MorganRO (2004) The annexins. Genome Biol 5: 219.1505925210.1186/gb-2004-5-4-219PMC395778

[45] RojasE, PollardHB, HaiglerHT, ParraC, BurnsAL (1990) Calcium-activated endonexin II forms calcium channels across acidic phospholipid bilayer membranes. J Biol Chem 265: 21207–21215.2174439

[46] FariaD, DahimèneS, AlessioL, Scott-WardT, SchreiberR, et al (2011) Effect of Annexin A5 on CFTR: regulated traffic or scaffolding? Mol Membr Biol. 28(1): 14–29.10.3109/09687688.2010.50626421067452

[47] BorthwickLA, BothaP, VerdonB, BrodlieMJ, GardnerA, et al (2011) Is CFTR-delF508 really absent from the apical membrane of the airway epithelium? PLoS One 6(8): e23226.2182624110.1371/journal.pone.0023226PMC3149652

[48] KakarSS, JennesL (1995) Expression of gonadotropin-releasing hormone and gonadotropin-releasing hormone receptor mRNAs in various non-reproductive human tissues. Cancer Lett. 98(1): 57–62.8529206

[49] TievaA, StattinP, WikströmP, BerghA, DamberJE (2001) Gonadotropin-releasing hormone receptor expression in the human prostate. Prostate 47(4): 276–284.1139817510.1002/pros.1072

[50] KoushikK, BandiN, SundaramS, KompellaUB (2004) Evidence for LHRH-Receptor Expression in Human Airway Epithelial (Calu-3) Cells and Its Role in the Transport of a LHRH Agonist. Pharmaceutical Research 21(6): 1034–1046.1521217010.1023/b:pham.0000029294.70707.74

[51] ReutelingspergerCP, van HeerdeW, HauptmannR, MaassenC, van GoolRG, et al (1994) Differential tissue expression of Annexin VIII in human. FEBS Lett. 349(1): 120–124.10.1016/0014-5793(94)00559-18045287

[52] KawaminamiM, TsuchiyamaY, SaitoS, KatayamaM, KurusuS, et al (2002) Gonadotropin-releasing hormone stimulates annexin 5 messenger ribonucleic acid expression in the anterior pituitary cells. Biochem Biophys Res Commun. 291(4): 915–920.10.1006/bbrc.2002.657311866452

[53] AlzamoraR, KingJDJr, HallowsKR (2011) CFTR regulation by phosphorylation. Methods Mol Biol. 741: 471–488.10.1007/978-1-61779-117-8_2921594802

[54] Baudouin-LegrosM, HinzpeterA, JaulmesA, BrouillardF, CostesB, et al (2005) Cell-specific posttranscriptional regulation of CFTR gene expression via influence of MAPK cascades on 3′UTR part of transcripts. Am J Physiol Cell Physiol 289(5): C1240–C1250.1594420610.1152/ajpcell.00595.2004

[55] Rowe SM. VerkmanAS (2013) Cystic fibrosis transmembrane regulator correctors and potentiators. Cold Spring Harb Perspect Med. 3(7): a009761.10.1101/cshperspect.a009761PMC368587923818513

